The article "Investigation of the Effects of Adhesive Materials of Different Types and Thicknesses on Dental Tissue Stress via FEM Analysis" was published in 2022. Journal: Biomed Res Int.

# Investigation of the Effects of Adhesive Materials of Different Types and Thicknesses on Dental Tissue Stress via FEM Analysis

**DOI:** 10.1155/2022/8493909

**Published:** 2022-07-23

**Authors:** Hakan Yasin Gönder, Reza Mohammadi, Abdulkadir Harmankaya, İbrahim Burak Yüksel, Didem Seda Gültekin

**Affiliations:** ^1^Department of Restorative Dentistry, Faculty of Dentistry, Necmettin Erbakan University, Baglarbasi Street No:4 Meram Konya, Turkey; ^2^Faculty of Dentistry, Necmettin Erbakan University, Baglarbasi Street No:4 Meram Konya, Turkey; ^3^Department of Oral Diagnose and Radiology, Faculty of Dentistry, Necmettin Erbakan University, Baglarbasi Street No:4 Meram Konya, Turkey; ^4^Beyhekim Oral and Dental Health Center, İhsaniye Mh. Abdul Ezel Paşa Cd. No:28 Pk.42040 Selçuklu Konya, Turkey

## Abstract

The aim of this study was to investigate the types and thicknesses of adhesive materials used in restorative treatment in dentistry in class I occlusal and class II disto-occlusal cavities and to examine the effects of stress distribution on enamel, dentin, restoration material, and adhesive material using the finite element stress analysis method. A 3-dimensional geometry of the tooth was obtained by scanning the extracted 26 numbered upper molar tooth with dental tomography. The 3D geometry obtained by using the Geomagic Design X 2020.0 software was divided into surfaces, and necessary arrangements were made. With the Solidworks 2013 software, 2 different cavity modeling, class I occlusal and class II disto-occlusal, with a cavity angle of 95 degrees on the 3D model, as well as 10, 30, and 50 micrometers thick, four types of adhesive materials and the modeling of the bulk-fill composite material on it were made. With finite element stress analysis, the stress distribution was analyzed using the Abaqus software. The materials used in the study are included in the simulation as isotropic linear elastic. Periodontal ligament and jawbone were not included in the analysis. A total of 600 N pressure was applied on the models. In our study, it was observed that the amount of stress on the tooth structures changed when the thickness, elastic modulus, and Poisson ratios of the adhesive material were changed. In addition, when all models are examined, it is seen that when the thickness is increased, more stress is placed on the adhesive material compared to the restoration, while when 50-micrometer-thick adhesive material is used, more stress is placed on the restoration compared to the adhesive material.

## 1. Introduction

Dental caries is one of the most common chronic diseases worldwide, one to which people are susceptible throughout their lives [1, 2]. Restorations mean changing the natural tooth biomechanical balance. This is especially true for resin-based composite restorations because the hardness of the materials used may not exactly match natural teeth [3].

The article "Investigation of the Effects of Adhesive Materials of Different Types and Thicknesses on Dental Tissue Stress via FEM Analysis" was published in 2022. Journal: Biomed Res Int.

Resin-based composites have been a revolutionary innovation in restorative materials. These materials were mainly developed to restore the aesthetics and function of teeth and are now widely used for class I and II restorations [4–6]. In particular, following the detailed examination and analysis of the forces occurring in the mouth, the forces emerging as a result of these analyses should be distributed according to an appropriate physiological balance, and the restorations on the teeth should be in accordance with the principles of oral rehabilitation [7]. The primary source of stress in a restored tooth is usually dimensional changes or occlusal loads at the interface of the composite, tooth, and restorative material [8].

This analysis method has been developed as a solution to certain problems that arise in experimental environments and are very difficult to solve. In this method, the object or material to be examined is modeled by dividing it into certain quantities of elements, and analyses are performed on these modeled parts. With the finite element method, some problems such as heat transfer, stress analysis, electromagnetism, and fluid mechanics can be analyzed [9–12]. Since this analysis method has many useful features, it has frequently been a preferred method for research in today's dentistry. While it is impossible to repeat a study many times in clinical trials, the experiments performed with this method can be easily repeated [13–16]. The analysis of materials with irregular shapes, which are used in many treatments in the field of dentistry, can be easily done with the finite element stress analysis method [17, 18].

This method is one of the most important modern scientific techniques, and the use of computer programs is mandatory as billions of arithmetic operations are performed in its application [7, 19]. Compared to laboratory tests, this analysis method has many advantages; living tissues are not needed and variables can be manipulated, while maximum standardization is achieved as a result [9]. Another advantage is that it is much less time-consuming compared to many other methods [14].

A warm air blow technique, an active application technique, and a double-layer application have been reported to improve the bonding performance of adhesive materials, and some of these techniques also influence the thickness of the adhesive layer [20–25]. The aim of this study was to investigate the types and thicknesses of adhesive materials used in restorative treatment in dentistry in class I occlusal and class II disto-occlusal cavities, as well as to examine the effects of stress distribution on enamel, dentin, restoration material, and adhesive material using the finite element stress analysis method.

The article "Investigation of the Effects of Adhesive Materials of Different Types and Thicknesses on Dental Tissue Stress via FEM Analysis" was published in 2022. Journal: Biomed Res Int.

## 2. Materials and Methods

The 3D geometry of tooth number 26, which was taken with a dental tomography [DA1] device, was scanned. Cone beam computerized tomography (CBCT) was taken using Morita 3D Accuitomo 170 (J Morita Mfg. Corp., Kyoto, Japan). The size of the imaging volume was a cylinder with diameter 40 × height 40 mm at the X-ray rotational center. Images were taken under the exposure condition of 90 kVp (X-ray tube voltage) and 5 mA (value of the electric current) which were the standard parameters and can be changed for different subjects. Images were taken using 160 qm and 17.5-second exposure time parameters. The 3D geometry created using the Geomagic Design X 2020.0 software was divided into surfaces, and necessary arrangements were made. Periodontal ligament (PDL) was not designed, so fixed and pinned boundary conditioning was used to simulate roots as fixed in the bone. The tooth model was placed in the coordinate system so that the *x*-axis defines the buccolingual direction, the *y*-axis defines the mesiodistal direction, and the *z*-axis is oriented upwards (Figure 1).

With the Solidworks 2013 software (Solidworks Corp., USA), two different cavities were modeled, class I occlusal and class II disto-occlusal, with a cavity angle of 95 degrees on the 3D model. A class I cavity with an occlusal depth of 4 mm and an occlusal-gingival depth (Figure 2). A class II cavity with an occlusal depth of 4 mm and an occlusal-gingival depth of 6 mm was fixed with the occlusal margin in the enamel and the gingival margin in dentin (Figure 3).

Since the elastic modulus and Poisson ratio of adhesive materials affect the stress values on dental tissues, restoration, and adhesive material, we chose adhesive materials with different elastic modulus and Poisson ratios in this study. Four types of adhesive material, of 10-, 30-, and 50-micrometer thicknesses (Table 1), were applied to the cavities. Afterwards, bulk-fill composite material was applied on the adhesive material.

With the finite element stress analysis method, the stress distribution was examined with the help of the Abaqus software (2020 Dassault Systems Simulation Corp., Johnston, RI, USA). The restorative materials used in our study were included in the simulation as isotropic linear elastic. Periodontal ligament and jawbone were not included in the analysis, and a total pressure of 600 N was applied on the models (Figure 1).

The article "Investigation of the Effects of Adhesive Materials of Different Types and Thicknesses on Dental Tissue Stress via FEM Analysis" was published in 2022. Journal: Biomed Res Int.

The total number of nodes of cavity models with different adhesive thicknesses is shown in Table 2.

## 3. Results

As a result of the change in the adhesive material thickness in all cavity models, the enamel and dentin thicknesses are constant, while the restoration thicknesses change. The thickness of the restoration decreases when the thickness of the adhesive material increases, and the thickness of the restoration increases when the thickness of the adhesive material decreases, but the enamel and dentin thicknesses remain constant in all models.

When all models are examined individually, while the thickness increases, more stress is placed on the adhesive material compared to the restoration, while when 50-micrometer-thick adhesive material is used, more stress is placed on the restoration compared to the adhesive material. In addition, when all models are considered, the stress values on the enamel and dentin were higher than the stress values on the restoration and adhesive material.

### 3.1. Results Obtained in Class I Cavity as a Result of Stress Analysis

When adhesive materials with either an elastic modulus of 3.6 GPa and a Poisson ratio of 0.28 or an elastic modulus of 1.9 GPa and a Poisson ratio of 0.28 (adhesive system 1 and adhesive system 2, respectively) and when the thickness of the class I occlusal cavity increases, the stress on the enamel and dentin increases, while the amount of stress on the restoration and adhesive material decreases. However, the highest stress value (Pmax) for enamel and dentin was found when 30-micrometer-thick adhesive material was used (Figures 4 and 5).

When an adhesive material with an elastic modulus of 1 GPa and a Poisson ratio of 0.3 (adhesive system 3) is used and when the thickness of the class I occlusal cavity increases, the stress on the enamel, dentin, and adhesive material decreases, while the amount of stress on the restoration increases. The highest stress value for enamel and dentin was found when 10-micrometer-thick adhesive material was used. Minimal changes were observed in the stresses on the dentin when 30-micrometer- and 50-micrometer-thick adhesive materials were used (Figure 6).

When an adhesive material with an elastic modulus of 1 GPa and a Poisson ratio of 0.24 (adhesive system 4) is used and when the thickness of the class I occlusal cavity increases, the stress on the enamel, dentin, and adhesive material decreases, while the amount of stress on the restoration material increases. However, when 50-micrometer-thick adhesive material was used, the amount of stress on the dentin increased slightly compared to the use of 30-micrometer-thick adhesive material. The highest stress value for enamel and dentin was found when 10-micrometer-thick adhesive material was used (Figure 7).

The article "Investigation of the Effects of Adhesive Materials of Different Types and Thicknesses on Dental Tissue Stress via FEM Analysis" was published in 2022. Journal: Biomed Res Int.

In class I occlusal cavity, when the elastic modulus is reduced from 3.6 GPa to 1.9 GPa while the Poisson ratio is constant and when 10-micrometer-thick adhesive material was used, no change was observed in the stresses on the enamel. When 30-micrometer-thick adhesive material is used, the stress on the enamel increases, while when 50-micrometer-thick adhesive material is used, the stress on the enamel decreases. On the other hand, when 10-, 30-, and 50-micrometer-thick adhesive materials are used on dentin, the stress values on the dentin increase. The stresses on the restoration increased when 10- and 30-micrometer-thick adhesive materials were used, while the stresses on the restoration decreased when 50-micrometer-thick adhesive material was used. The stresses on the adhesive material decreased when 10-, 30-, and 50-micrometer-thick adhesive materials were used (Figure 8).

In class I occlusal cavity, when the elastic modulus is constant and the Poisson ratio is reduced from 0.3 to 0.24 and while the amount of stress on enamel decreased when 10-micrometer-thick adhesive material was used, the stress on enamel increased when 30- and 50-micrometer-thick adhesive material was used. On the other hand, the amount of stress on dentin did not change when 10-micrometer-thick adhesive material was used, while the stress on dentin increased when 30- and 50-micrometer-thick adhesive materials were used. Stress on restoration decreased when 30-micrometer-thick adhesive material was used but increased when 10- and 50-micrometer-thick adhesive materials were used. The stresses on the adhesive material decreased when 10-, 30-, and 50-micrometer-thick adhesive materials were used (Figure 9).

### 3.2. Results Obtained in Class II Cavity as a Result of Stress Analysis

When an adhesive material with an elastic modulus of 3.6 GPa and a Poisson ratio of 0.28 (adhesive system 1) is used, the highest stress value in the enamel in the class II disto-occlusal cavity occurs when an adhesive material with a thickness of 50 micrometers is used, while the lowest amount of stress occurs when an adhesive material with a thickness of 30 micrometers is used. In dentin, on the other hand, the highest stress value occurs when an adhesive material with a thickness of 30 micrometers is used, while the lowest amount of stress occurs when an adhesive material with a thickness of 10 micrometers is used. The amount of stress on the restoration and adhesive material decreases as the thickness increases (Figure 10).

When an adhesive material with an elastic modulus of 1.9 GPa and a Poisson ratio of 0.28 (adhesive system 2) is used, the highest stress value in the enamel in the class II disto-occlusal cavity occurs when 50-micrometer-thick adhesive material is used, while the lowest amount of stress occurs when an adhesive material with a thickness of 30 micrometers is used. In dentin, on the other hand, the highest stress value occurs when an adhesive material with a thickness of 30 micrometers is used, while the lowest amount of stress occurs when an adhesive material with a thickness of 10 micrometers is used. The amount of stress on the restoration and adhesive material decreases as the thickness increases (Figure 11).

The article "Investigation of the Effects of Adhesive Materials of Different Types and Thicknesses on Dental Tissue Stress via FEM Analysis" was published in 2022. Journal: Biomed Res Int.

When an adhesive material with an elastic modulus of 1 GPa and a Poisson ratio of 0.3 (adhesive system 3) is used, the highest stress value in the enamel in the class II disto-occlusal cavity occurs when an adhesive material with a thickness of 50 micrometers is used, while the lowest amount of stress occurs when an adhesive material with a thickness of 30 micrometers is used. In dentin, on the other hand, the highest stress value occurs when an adhesive material with a thickness of 30 micrometers is used, while the lowest amount of stress occurs when an adhesive material with a thickness of 10 micrometers is used. The amount of stress on the restoration and adhesive material decreases as the thickness increases (Figure 12).

When an adhesive material with an elastic modulus of 1 GPa and a Poisson ratio of 0.24 (adhesive system 4) is used, the highest stress value in the enamel in the class II disto-occlusal cavity occurs when 50-micrometer-thick adhesive material is used, while the lowest amount of stress occurs when 30- and 10-micrometer-thick adhesive materials are used. In addition, when 10- and 30-micrometer-thick adhesive materials were used, no change was observed in the stresses on the enamel. In dentin, on the other hand, the highest stress value occurs when using adhesive material with a thickness of 30 micrometers, while the lowest amount of stress occurs when using adhesive material with a thickness of 10 micrometers. The amount of stress on the restoration and adhesive material decreases as the thickness increases (Figure 13).

When the elastic modulus is reduced from 3.6 GPa to 1.9 GPa while the Poisson ratio is constant in the class II disto-occlusal cavity, the amount of stress on enamel and dentin increased when 10-, 30-, and 50-micrometer-thick adhesive materials were used. The amount of stress on the restoration increased when 10- and 50-micrometer-thick adhesive materials were used but decreased when 30-micrometer-thick adhesive material was used. The stresses on the adhesive material decreased when 10-, 30-, and 50-micrometer-thick adhesive materials were used, and the greatest rate of reduction in stress occurred when adhesive material with a thickness of 10 micrometers was used (Figure 14).

The article "Investigation of the Effects of Adhesive Materials of Different Types and Thicknesses on Dental Tissue Stress via FEM Analysis" was published in 2022. Journal: Biomed Res Int.

In class II disto-occlusal cavity, when the elastic modulus is constant and the Poisson ratio is reduced from 0.3 to 0.24, the amount of stress on enamel and dentin increased when 10-, 30-, and 50-micrometer-thick adhesive materials were used. The stress values on restoration and adhesive material decreased when 10-, 30-, and 50-micrometer-thick adhesive materials were used (Figure 15).

## 4. Discussion

Knowing the intraoral biomechanics, the stresses caused by the forces on the teeth and their destructive effects on the dental tissues ensure that the restorations are more successful and long lasting.

Meijer et al. in their study proved that the two-dimensional analysis does not reflect reality sufficiently [32]. In other studies, it has been shown that the three-dimensional finite element stress analysis method gives more realistic results [33–35]. In addition, Kamposiora et al. stated that the method would be simpler by reducing the three-dimensional material data to two dimensions, so that high-capacity computers would not be needed and the cost would be reduced [36].

Directly applied posterior resin composites, machinable block composites, and ceramic materials can be used successfully to restore decayed teeth [37]. These materials are able to resist the occlusal forces of class I and II restorations. Direct or indirect restorative materials and technologies are widely used; however, there is no consensus on the best choice for restoration [38]. We used bulk-fill composite as restorative material in our study. Bulk-fill composites can be adequately polymerized at a thickness of 4 mm [39–41]. Some studies showed a possible depth of cure up to 5.5 mm [42]. Further, bulk-fill composites result in having less shrinkage and lower values of contraction stress in comparison to the conventional types of composite resins [43]. It has been suggested that it may be beneficial to use a thin layer of restorative materials such as glass ionomer cements, flowable composites, or nanofilled adhesives into the cavity before resin filling materials are applied to reduce stress [44]. The stiffness or elastic modulus of dental restorative materials and adhesive materials is extremely important at the adhesive-tooth-restoration interface. Ausiello et al. showed that in class II adhesive restorations, tubercle displacement is greater for more rigid composites due to stress from polymerization shrinkage, but lower tubercle movements are seen when more flexible composites are used [45].

The article "Investigation of the Effects of Adhesive Materials of Different Types and Thicknesses on Dental Tissue Stress via FEM Analysis" was published in 2022. Journal: Biomed Res Int.

In the literature, there are studies using different adhesive thicknesses such as 2, 5, 10, and 30 micrometers. In the study by Ausiello et al. in 2011, a thin (10 micrometers) adhesive layer was used [46]. The thicker the adhesive layer, the higher the magnitude of the peel stresses and strains and thus the larger the bending deformation [47]. Takamizawa et al. in their study changed the adhesive thickness clinically by applying strong or light air to the adhesive material, increasing or decreasing the air application time, and applying the adhesive material in layers [48].

Alp et al. prepared three class II models using an adhesive layer with a thickness of 30 micrometers [49]. In the first model, amalgam (M1) was placed on the adhesive and in the second model glass carbomer cement (M2), and in the third model, 1 mm thick resin modified glass ionomer cement was placed on it, followed by a 30-micrometer-thick adhesive material and then resin composite (M3). While the stress values occurring in the adhesive layer as a result of the forces applied to the models were close and high in the M2 and M3 models, the lowest value was found in the M1 model. At the same time, when the stress values in all models were examined in this study, it was observed that more stress occurred in the restoration materials and adhesive material compared to enamel and dentin.

Kemp-Scholte and Davidson, in their study in 1990, reported that the thicker adhesive layer caused the formation of lower interface stresses [44]. A greater adhesive layer thickness can theoretically be beneficial in terms of providing a more flexible and stress-absorbing transition between dentin and composite [50].

In the study by Coelho et al., which uses the three-dimensional finite element stress analysis method, it was observed that the maximum stress values increased and the bond strength values decreased as the adhesive thickness increased for single bond [50]. In a study by Zheng et al., it was reported that the bond strength decreases as the adhesive layer thickness increases for single bond [51]. In our study, when the adhesive system with a Poisson ratio of 0.28 and an elastic modulus of 3.6 GPa, or a Poisson ratio of 0.28 and an elastic modulus of 1.9 GPa, is used in class I occlusal cavity, the stresses on enamel and dentin are low when 10-micrometer-thick adhesive material is used, while it increases when 30-micrometer-thick adhesive material is used. However, when the adhesive thickness was increased to 50 micrometers, the stress values on enamel and dentin decreased again. As a result, the clinical benefits of having a thin or thick adhesive layer are still a matter of debate [52, 53].

The article "Investigation of the Effects of Adhesive Materials of Different Types and Thicknesses on Dental Tissue Stress via FEM Analysis" was published in 2022. Journal: Biomed Res Int.

## 5. Conclusion

Elastic modulus, Poisson ratio, and thickness of the adhesive material are used in restorative dentistry. It significantly affects the amount of stress on the enamel, dentin, restorative material, and adhesive material. For adhesive materials and composites of different hardness, FEM analysis allows the determination of the optimum adhesive layer thickness that provides maximum stress distribution. However, there are not enough studies in the literature on the effects of the thickness of the adhesive materials on the stresses on dental tissue.

In our study, when the elastic modulus decreases while the Poisson ratio remains constant, the stress values on enamel and dentin in class I and class II cavities vary, but the thickness of the adhesive material, where the maximum stresses occur, did not change. Also, when the elastic modulus is constant and the Poisson ratio decreases, the stress values on enamel and dentin in class I and class II cavities show a slight variation, while the thickness of the adhesive material at which the maximum stresses occur does not change. When all models are examined individually, while the thickness increases, more stress is placed on the adhesive material compared to the restoration, while when 50-micrometer-thick adhesive material is used, more stress is placed on the restoration compared to the adhesive material. At the same time, it was found in our study that the stress values on the enamel and dentin in all models were higher than the stress values on the restoration and adhesive material.

## Figures and Tables

**Figure 1:** Load and boundary conditions.

**Figure 2:** (a) Buccolingual cross-section of the restored tooth. (b) Class I occlusal cavity. (c) Adhesive layer. (d) Dentin. (e) Restoration. (f) Enamel. (g) Pulp.

**Figure 3:** Class II disto-occlusal cavity. (a) Adhesive layer. (b) Dentin. (c) Enamel. (d) Pulp. (e) Restoration.

**Figure 4:** Stress distribution regions in a tooth with a class I occlusal cavity when using adhesive system 1 with a thickness of 10, 30, and 50 micrometers, respectively.

**Figure 5:** Stress distribution regions in a tooth with a class I occlusal cavity when using adhesive system 2 with a thickness of 10, 30, and 50 micrometers, respectively.

**Figure 6:** Stress distribution regions in a tooth with a class I occlusal cavity when using adhesive system 3 with a thickness of 10, 30, and 50 micrometers, respectively.

**Figure 7:** Stress distribution regions in a tooth with a class I occlusal cavity when using adhesive system 4 with a thickness of 10, 30, and 50 micrometers, respectively.

**Figure 8:** Class I occlusal cavity with elastic modulus reduced from 3.6 GPa to 1.9 GPa with fixed Poisson's ratio.

The article "Investigation of the Effects of Adhesive Materials of Different Types and Thicknesses on Dental Tissue Stress via FEM Analysis" was published in 2022. Journal: Biomed Res Int.

**Figure 9:** Class I occlusal cavity with Poisson ratio reduced from 0.3 to 0.24 with fixed elastic modulus.

**Figure 10:** Stress distribution regions in a tooth with a class II disto-occlusal cavity when using adhesive system 1 with a thickness of 10, 30, and 50 micrometers, respectively.

**Figure 11:** Stress distribution regions in a tooth with a class II disto-occlusal cavity when using adhesive system 2 with a thickness of 10, 30, and 50 micrometers, respectively.

**Figure 12:** Stress distribution regions in a tooth with a class II disto-occlusal cavity when using adhesive system 3 with a thickness of 10, 30, and 50 micrometers, respectively.

**Figure 13:** Stress distribution regions in a tooth with a class II disto-occlusal cavity when using adhesive system 4 with a thickness of 10, 30, and 50 micrometers, respectively.

**Figure 14:** Class II disto-occlusal cavity with elastic modulus reduced from 3.6 GPa to 1.9 GPa with fixed Poisson's ratio.

**Figure 15:** Class II disto-occlusal cavity with Poisson ratio reduced from 0.3 to 0.24 with fixed elastic modulus.

**Table 1:** Mechanical properties of structures used in 3D finite element stress analysis models of maxillary molars.

Material	Elastic modulus	Poisson's ratio	Tensile strength	Compressive strength	
Dentin	18.6 GPa [26]	0.31 [26]	98.7 MPa [27]	297.0 MPa [27]	
Enamel	84.1 GPa [26]	0.33 [26]	10.3 MPa [27]	384.0 MPa [27]	
Pulp	0.002 GPa [28]	0.45 [28]	—	—	
Bulk-fill composite	12.0 GPa [29]	0.25 [29]	42 MPa [27]	169.0 MPa [27]	
Adhesive system 1	3.6 GPa [30]	0.28 [30]	—	—	
Adhesive system 2	1.9 GPa [30]	0.28 [30]	—	—	
Adhesive system 3	1 GPa [3]	0.3 [3]	—	—	
Adhesive system 4	1 GPa [31]	0.24 [31]	—	—	

**Table 2:** Total number of nodes of cavity models with different adhesive thicknesses. Mesh type of all models is linear tetrahedral elements of C3D4.

Model	Total nodes
Occlusal cavity with a 10-micrometer-thick adhesive material	1361383
Occlusal cavity with a 30-micrometer-thick adhesive material	1359713
Occlusal cavity with a 50-micrometer-thick adhesive material	1356435
Disto-occlusal cavity with a 10-micrometer-thick adhesive material	1368958
Disto-occlusal cavity with a 30-micrometer-thick adhesive material	1365634
Disto-occlusal cavity with a 50-micrometer-thick adhesive material	1365307

## Data Availability

No data were used in this study.
